The article "The Extracellular Matrix Glycoprotein Tenascin C and Adult Neurogenesis" was published in 2021. Journal: Front Cell Dev Biol.

# The Extracellular Matrix Glycoprotein Tenascin C and Adult Neurogenesis

**DOI:** 10.3389/fcell.2021.674199

**Published:** 2021-04-29

**Authors:** Milena Tucić, Vera Stamenković, Pavle Andjus

**Affiliations:** Center for Laser Microscopy, Institute for Physiology and Biochemistry “Jean Giaja”, Faculty of Biology, University of Belgrade, Belgrade, Serbia

**Keywords:** tenascin C, adult neurogenesis, subgranular zone, subventricular zone, astrocyte, microglia, stem cell migration

## Abstract

Tenascin C (TnC) is a glycoprotein highly expressed in the extracellular matrix (ECM) during development and in the adult central nervous system (CNS) in regions of active neurogenesis, where neuron development is a tightly regulated process orchestrated by extracellular matrix components. In addition, newborn cells also communicate with glial cells, astrocytes and microglia, indicating the importance of signal integration in adult neurogenesis. Although TnC has been recognized as an important molecule in the regulation of cell proliferation and migration, complete regulatory pathways still need to be elucidated. In this review we discuss the formation of new neurons in the adult hippocampus and the olfactory system with specific reference to TnC and its regulating functions in this process. Better understanding of the ECM signaling in the niche of the CNS will have significant implications for regenerative therapies.

## Introduction

In contrast to the main form of neural plasticity inferring modifications at the synaptic level, adult neurogenesis confers plasticity through the addition of a population of newly developed neurons with functional synaptic inputs and outputs. Production of new neurons continues throughout life in most invertebrate and vertebrate species even after fetal and early postnatal development has ceased (Cayre et al., 2002). In the adult human brain neurogenesis remains a controversial area of research with evidence both for and against a significant rate of production of new neurons (Eriksson et al., 1998; Spalding et al., 2013; Sorrells et al., 2018). The fact that it is evolutionarily conserved implies that adult neurogenesis is of great functional importance. Nevertheless, adult neurogenesis is restricted to the dentate gyrus (DG) of the hippocampus and the subventricular zone (SVZ) around lateral ventricles (LV) (Altman and Das, 1965; Altman, 1969). Arguably, adult neurogenesis may also happen in other regions (Bernier et al., 2002; Zhao et al., 2003). However, the two established neurogenic niches, the SVZ and the hippocampus, are residential areas for neural stem cells (NSC) where tightly regulated processes of neuronal development are orchestrated by extracellular matrix (ECM) components. In addition, newborn cells also communicate with glia, underlining signal integration in adult neurogenesis.

Tenascin C (TnC) is a member of the tenascin family, comprised of glycoproteins highly expressed in the ECM during development and in the adult central nervous system (CNS) in regions of active neurogenesis (Bartsch et al., 1992; Gates et al., 1995; Ferhat et al., 1996). The term tenascin is derived from the Latin words *tenere*—to hold, and *nasci*—to be born, referring to the presence of tenascins in fetal tissue (Chiquet-Ehrismann et al., 1986). Nowadays, it is known that TnC is involved in morphogenic changes during development and tissue remodeling, as well as in cell adhesion and signaling between cells (Jones and Jones, 2000).

In order to understand the functional significance of adult neurogenesis, we need to elucidate the circumstances that modulate the process of addition of newborn neurons into the brain. Most of the research is focused on neurons, while the influence of non-neuronal cells and the ECM are less considered although they both provide stimuli that lead the processes of neurogenesis. Growing body of research points to the importance of glial cells and the ECM in the understanding of cellular plasticity. Thus, in this review we discuss the formation of new neurons in the adult hippocampus and the olfactory system in rodent animal models with specific reference to TnC and its regulating functions in this process. Although direct evidence regarding the role of TnC in processes of adult neurogenesis is lacking, its functions found in other contexts could be extrapolated to adult neurogenesis as potentially important.

## General Features of Adult Neurogenesis

New neurons are generated from NSC, a population of self-renewing, multipotent cells. Through the process of self-renewal, a constant pool of dividing cells can be maintained, and the potential of NSC to differentiate into diverse cell types allows for the creation of new neurons and astrocytes. Under physiological conditions NSC can be found in the SVZ surrounding the LV, from where newborn cells migrate to the olfactory bulb (OB), and in the subgranular zone (SGZ) of the DG, where new cells become functionally integrated into existing neuronal circuits. The processes of proliferation, migration and differentiation in the two niches have different spatial and temporal organizations, while the addition of new synapses in an activity dependent manner is under control of neural activity (Ma et al., 2009).

Adult hippocampal neurogenesis is found to be confined to the DG. Namely, local radial glial stem cells in the SGZ undergo proliferation and through asymmetric division give rise to neurons or astrocytes (Kriegstein and Alvarez-Buylla, 2009). The daughter cells originating from the radial glial stem cells are highly proliferative amplifying stem cells, which in turn generates neuroblasts (Gonçalves et al., 2016). New immature neurons show limited migration from the SGZ to the granular cell layer (GCL). Four weeks after proliferation, they begin to express markers of mature neurons (Kempermann et al., 2003). Most of the newborn neurons in the hippocampus differentiate into excitatory granular cells, although there is also a detectable number of newborn interneurons (Liu et al., 2003). After the maturation phase, newborn neurons are indistinguishable from the neighboring mature neurons when characterized by electrical and synaptic properties (Ge et al., 2007).

In contrast to the events during adult hippocampal neurogenesis, newborn cells in the SVZ migrate a long distance to the OB (Alvarez-Buylla and Garcìa-Verdugo, 2002). After proliferation at the stage of neuroblasts, residing cells follow the chain of migration along the rostral migratory stream (RMS) generated by specialized astrocytes. Upon reaching the middle of the OB, cells in the stage of immature neurons detach from the chain and continue to perform radial migration. This is followed by differentiation into two types of interneurons. Most of them differentiate into GABAergic granular neurons, while the rest become periglomerular neurons expressing GABA and/or dopamine as neurotransmitters. Complete integration of newborn neurons into existing circuits requires the establishment of both synaptic inputs and outputs, in order for them to be able to receive and respond to olfactory stimuli (Bonzano et al., 2016).

## Tenascin C: Expression, Structure, Interactions

Matricellular proteins are a group of proteins that are secreted into the ECM but do not have a primary role in the maintenance of its structure (Bornstein, 2009). The term was introduced to explain the diversity of functions of proteins such as TnC. TnC is a glycoprotein present in the ECM as a regulatory protein with different spatial and temporal expression patterns during life. In fact, it is widespread during development, while its expression decreases during life, and remains restricted to plastic areas of active neurogenesis (Gates et al., 1995; Ferhat et al., 1996). In addition, TnC was found to be expressed *de novo* in lesions and during wound healing (Roll and Faissner, 2019), but also in pathological conditions, such as inflammation, cancer and trauma (Chiquet-Ehrismann and Chiquet, 2003; Midwood et al., 2011). During CNS development TnC is expressed by radial glial cells (Götz et al., 1997), while in the adult CNS, TnC is produced by astrocytes in the SVZ (Kazanis et al., 2007) and granule cells in the hippocampus (Niquet et al., 1995).

In development, disease and regeneration the TnC gene is regulated through cytokines, growth factors and mechanical stimuli (Chiovaro et al., 2015). The expression of TnC during embryogenesis is often associated with morphogenetic changes by mechanisms of segmentation and gene patterning. A number of pro- and anti-inflammatory cytokines has been shown to induce expression of TnC in different cell types, although so far there were no related functional studies. Control of TnC promoter activity is also achieved through upstream regulation by the platelet-derived growth factor and the transforming growth factor-β. Transduction of external mechanical stimuli results in increased TnC expression by way of the activation of the Rho/ROCK signaling cascade that activates the TnC promoter. TnC becomes a functional protein after post-transcriptional and post-translational modifications, such as gene splicing and protein glycosylation (Giblin and Midwood, 2015). Export and incorporation of the suitably modified protein into the ECM is dependent on the ECM composition, while the expression of TnC in different tissues is regulated through proteolytic degradation.

TnC is a hexamer, each monomer consisting of the tenascin assembly (TA) domains at the N-terminus, responsible for the assembly of oligomeric proteins, epidermal growth factor-like (EGFL) repeats, fibronectin type III (FN III) domains, and a globular fibrinogen domain at the C-terminus (Figure 1A). Alternative splicing within the FN III domains allows for different isoforms of TnC. Multidomain structure of TnC allows for a variety of interactions with components of the ECM and different types of cells (Midwood et al., 2016). It was first recognized as a molecule that participates in cell adhesion, while later studies suggested that it regulates cell signaling, migration and differentiation (Chiquet-Ehrismann et al., 1986). TnC is engaged in the regulation of cell migration since it is able to perform both adhesive and anti-adhesive interactions (Figure 1B; Faissner and Kruse, 1990; Lochter and Schachner, 1993). TnC is able to influence cell behavior through direct interactions with cell surface receptors, including integrins (Schnapp et al., 1995; Yokosaki et al., 1998), but also with ECM components, fibronectin and chondroitin-sulfate proteoglycans, such as phosphacan (Figure 2; Milev et al., 1997; Jones and Jones, 2000).

**FIGURE 1:** The structure of human tenascin C and its involvement in different regulatory pathways. **(A)** Schematic representation of a TnC monomer composed of N-terminal tenascin assembly (TA) domain, epidermal growth factor-like (EGFL) repeats, two types of fibronectin III (FN III) domains, constitutively expressed domains in TnC variants and alternatively spliced domains, and the C-terminal fibrinogen globe. **(B)** TnC as a functional hexamer participates in processes of cell proliferation, adhesion, migration, differentiation, cell survival and apoptosis, synaptic functions and in the inflammatory response.

**FIGURE 2:** Schematic representation of TnC interactions with cell surface receptors and extracellular matrix components. Signaling from epidermal growth factor (EGF), integrins, Toll-like receptor 4 (TLR4) and Wnt to intracellular effectors such as focal adhesion kinase (FAK), mitogen-activated protein kinase (MAPK), phospholipase C (PLC), leads to changes in gene transcription, resulting in changes of expression of proteins involved in proliferation, adhesion, cell survival/apoptosis, synaptic activity and immune response. TnC performs interactions with components of ECM collagen, fibronectin and chondroitin-sulfate proteoglycans, such as phosphacan, a short form of receptor protein tyrosin phosphatase β.

Although TnC is a crucial regulatory molecule during development and organogenesis, TnC deficient mice are able to develop normally (Saga et al., 1992). However, after morphological and electrophysiological changes in TnC deficient mice have been documented (Evers et al., 2002; Irintchev et al., 2005), it has been demonstrated that TnC deficiency leads to behavioral abnormalities as well (Morellini and Schachner, 2006). Moreover, a detailed study confirmed these results and suggested how TnC interacts with the environment in shaping the behavioral phenotype (Stamenkovic et al., 2017a).

### Tenascin C in the Adult Stem Cell Niche

The stem cell niche is a microenvironment where stem cells reside and receive signals that determine their fate. A myriad of signals affects stem cell behavior, including signals from the neighboring cells and the ECM, making cell-to-cell and cell-to-matrix interactions determine whether the cells stay in quiescent state or begin to proliferate. In the SGZ, the thin lamina between the hippocampal hilus and the granular cell layer, proliferating cells are found in clusters around small capillaries (Palmer et al., 2000). Proliferating cells can be labeled with bromodeoxyuridine (BrdU), a synthetic analog of thymidine which incorporates into the DNA during cell division. Cells positive for BrdU, also expressing endothelial markers, were found in this anatomical niche, suggesting that adult neurogenesis actually occurs within the angiogenic niche. In addition, in the SVZ, proliferating cells are located next to blood vessels, while quiescent cells are located adjacent to the epidermal layer lining the ventricles (Tavazoie et al., 2008; Morante-Redolat and Porlan, 2019).

In the adult murine brain along NSC, supporting cells and ECM components, the microenvironment of the neurogenic niche also contains specific proteins, such as TnC and thrombospondin (Garcion et al., 2001; Kazanis et al., 2007; Faissner et al., 2017). As a prominent component of the stem cell niche, TnC guides the processes of NSC development (Chiquet-Ehrismann et al., 2014). NSC have been identified as the main source of their local ECM, since single-cell RNA sequencing of quiescent NSC in the SVZ showed that these cells are rich in mRNA encoding for matrix proteins, while activated NSC or neuroblasts express very few ECM components (Kjell et al., 2020). In addition, proteome analysis showed an enrichment of TnC in the OB and SVZ, compared to the medial side of the lateral ventricle. Assessing the OB, an increase in stiffness was found from the SVZ and RMS toward the OB, implying that cell migration depends on tissue mechanobiology, as it was already known that biochemical and biophysical properties of NSC niche shape adult neurogenesis. Microelastic mapping of the rat DG has shown that ECM in the SGZ, where the population of progenitor cells reside, and the hilus, through which new axons extend to the CA3 region, have lower stiffness than the GCL, wherein differentiated cells migrate (Luque et al., 2016). This was in correspondence with earlier *in vitro* studies, where it was shown that stiffness regulates NSC differentiation. More precisely, soft ECM promotes NSC differentiation, while stiff ECM suppresses it (Saha et al., 2008). In addition, neurite outgrowth of the differentiating NSC is dependent on the stiffness of the growth medium (Stukel and Willits, 2018). Although it is clear that tissue stiffness correlates with cell density (Koser et al., 2015), niche-specific mechanical properties in both neurogenic areas can also be considered as a consequence of the presence of specific components of the proteome. Nevertheless, more detailed studies concerning the involvement of TnC in the mechanical properties of neurogenic niches could provide valuable information, considering its role in mechanotransduction and control of neurite outgrowth (Chiquet et al., 2007; Andrews et al., 2009).

Cell surface proteins, such as stretch-sensitive ion channels and integrins are able to sense mechanical forces and convert them into biochemical signals. FN III domains of TnC interact with different integrins (Tucker and Chiquet-Ehrismann, 2015) causing a rapid cytoskeleton response to external forces by Rho-dependent actin assembly and contraction (Asparuhova et al., 2009). As a consequence, a change in cell-matrix adhesion changes cell shape and orientation. In this way, the cell can continuously modify its response to external stimuli. Moreover, TnC expression can be induced by mechanical stress such as stretch in fibroblasts (Chiquet et al., 2007). The extensibility of the FN III domains (Oberhauser et al., 1998) imposes elastic properties to the TnC hexamer, directly contributing to tissue elasticity and protection against mechanical stress.

Since mechanical characteristics of the ECM, such as the grade of stiffness and elasticity, are involved in stem cell differentiation by means of affecting lineage commitment, this might be particularly important after tissue injury, where subsequent scar formation might negatively affect the ability of stem cells for repair.

### Cell Proliferation

When NSC receive the proper signal, they leave the quiescent state and begin to proliferate. Many extrinsic and intrinsic factors are involved, and TnC has been recognized as an important molecule in the regulation of NSC proliferation, which was first demonstrated in a study by Garcion and coworkers (Garcion et al., 2001). They showed that TnC knockout mice have reduced rates of proliferating cells in the SVZ, suggesting a supportive role of TnC in NSC proliferation. Another role for TnC was proposed by Garwood et al., who suggested the participation of TnC in differentiation of oligodendrocyte precursor cells (Garwood et al., 2004). They noticed a more rapid differentiation of cultured oligodendrocyte precursor cells in the absence of TnC. These two roles could be accomplished through the interaction with Sam68, a protein involved in the Src-like kinase apoptotic pathway. Furthermore, another study by Garcion and coworkers showed that TnC controls the fibroblast growth factor and epidermal growth factor responsiveness and differentiation properties of NSC (Garcion et al., 2004). This study confirmed the inhibitory effect of TnC on neurogenesis, and suggested that TnC deficient neurospheres had higher number of NSC that differentiated into neurons or glia. Moreover, another study showed an increased proliferation of astroglial progenitors in the spinal cord of TnC knockout mice during the embryonic period (Karus et al., 2011). On the other hand, mesenchymal stem cells are able to transdifferentiate into neural linages under specific conditions, and when grown on surface coated by TnC and tenascin R, they differentiate into neurons or oligodendrocytes (Tsai et al., 2014).

Intriguingly, in spite of the importance of TnC during embryonic and early postnatal NSC and neural progenitor proliferation and migration, it was demonstrated that TnC deficiency does not affect the number of NSC nor their progeny, neuroblasts, and periglomerular interneurons, in adult mice (Kazanis et al., 2007). Nevertheless, mice with TnC deficiency showed morphological changes around the LV that were reflected in an increased number of neuroblast clusters along the LV. The authors suggested a network of compensatory ECM molecules in the adult brain that are able to partially compensate for the loss of TnC.

Although some evidence about the role of TnC in cell proliferation is contradictory, there are a few regulatory mechanisms of proliferation involving TnC (Figure 2). EGFL repeats of TnC directly interact with the EGF receptor, activating the signaling pathways of phospholipase C, Ras/mitogen activated protein kinase (MAPK) and phosphatidylinositol 3-kinase (PI3)/Akt (Faissner et al., 2017; Hanmin et al., 2020). Proteomics-based research has also shown that TnC can be regulated by the modification of Human Natural Killer-1 (CD57) cells in NSC (Yagi et al., 2010). Namely, post-translational modification of CD57 stimulates TnC-dependent proliferation of NSC via the MAPK pathway. On the other hand, it has been shown that Sam68 is downregulated in cultured NSC in the presence of TnC, while increased expression of this splicing regulator causes a decrease in the proliferation of glial precursors (Moritz et al., 2008). A later study has shown that TnC interacts with lipid rafts in the oligodendrocyte membrane which leads to the inhibition of differentiation of these cells in culture (Czopka et al., 2010). In fact, TnC interferes with phosphorylation of Akt which in turn reduces expression of myelin basic protein and Sam68 in a PI3 kinase-dependent pathway. Also, there are indications that TnC regulates intracellular pathways via modulation of GTPase RhoA and focal adhesion kinase, leading to downstream modification of actin cytoskeleton (Midwood and Schwarzbauer, 2002). TnC disrupts intracellular localization of Rho, disabling its recruitment to the cell membrane. This event has the potential to evoke downstream modification of actin cytoskeleton that ends in the modifications of cell adhesion, contractility, cell cycle progression and gene transcription (Hall, 1998).

### Survival of Newborn Cells

Programmed cell death is considered to be a regulatory mechanism for maintaining the rate of experience-dependent adult neurogenesis. A decrease in BrdU-labeled cells in the adult SGZ has been reported, particularly in the first week of their life (Kempermann et al., 2004). The decrease in the number of proliferating BrdU-immunopositive cells is due to the programmed cell death by apoptosis (Biebl et al., 2000). This was later confirmed by Sierra et al. who showed that the majority of the amplifying progenitors undergo cell death by apoptosis during transition to neuroblasts (Sierra et al., 2010). These events take place in the first 4 days of their life and account for most of the decrease in neurogenic rate, this being considered as the main critical period of survival of newborn cells in the adult SGZ. Apoptosis is coupled to microglial phagocytosis, where newborn cells are engulfed by unchallenged microglia (Figure 3), with ramified morphology and low expression of typical inflammatory markers, such as CD11 and CD68, suggesting a non-inflammatory activation pathway. This was supported by the results on microglial transcriptomes that revealed the presence of non-inflammatory mediators in microglia in the developing and adult mouse brain (Bennett et al., 2016). Moreover, phagocytosis is not merely a passive removal of intracellular contents, but it also has an active role in maintaining neurogenesis. Microglia, through its secretome, provides a negative feedback loop, acting as a sensor for local cell death, modulating the balance between proliferation and survival of newborn cells. Thus, Diaz-Apacio et al. used a monolayer of neural progenitor cells derived from neurospheres to model neurogenesis, and allowed them to differentiate in the presence of conditioned medium from control and phagocytic microglia (Diaz-Aparicio et al., 2020). The results showed that the secretome of phagocytic microglia limits neurogenesis through the reduction in the production of neuronal-committed cells. To confirm these results, the hypothesis has been tested *in vivo*, following the injection of microglia conditioned medium in adult mice. The authors concluded that adult neurogenesis in the hippocampus is under a negative feedback loop provided by microglia. In contrast, a direct role of microglia in the regulation of newly generated neurons in the OB has not been reported.

**FIGURE 3:** Schematic representation of glial contribution to the regulation of adult neurogenesis. Astrocytes and microglia secrete growth factors and cytokines that guide the processes of neurogenesis. Microglia participates in the regulation of the neurogenic rate by engulfing apoptotic cells.

A wide range of microglial functions have been shown to be under TnC regulation during early postnatal development, among them cytokine/chemokine secretion, iNOS and COX2 expression, as well as chemotaxis and phagocytosis (Haage et al., 2019). The same study suggested that TnC controls microglial phagocytic activity via histone deacetylase, a protein that has already been linked to microglial functions. Involvement of TnC in microglial functions in CNS disorders has shown that TnC deficient mice have reduced microglial surveillance in the ischemic brain (Manrique-Castano et al., 2020).

In the adult brain, microglia is mostly studied for its role in the immune response, but there have been indications that microglia is involved in adult neurogenesis in a regulatory way, that includes some components of the inflammatory pathway. Brain inflammation has been shown to be detrimental for neurogenesis since activated microglia has a neurotoxic effect on newborn cells through release of IL-1, IL-6, nitric-oxide and reactive oxygen species (Valliéres et al., 2002). A negative correlation has been reported between the number of activated microglia in the rat hippocampus with the number of surviving new neurons (Figure 3; Ekdahl et al., 2003). In addition, the application of a selective inhibitor of microglial activation, minocycline, led to the restoration of hippocampal neurogenesis. There was no evidence that microglia suppresses cell proliferation or neuronal differentiation neither in basal nor in insult-induced neurogenesis.

Expression of TnC in areas of inflammation and tissue damage in inflamed rheumatoid joints suggests its involvement in inflammatory processes. It was shown on mice *in vivo* that TnC mediates joint inflammation by helping to maintain inflammation, although it does not seem to be involved in its initiation (Midwood et al., 2009). The same study showed that TnC induces synthesis of proinflammatory cytokines in human macrophages by the activation of Toll-like receptor 4 (TLR4). A later study that used experimental sepsis *in vivo* as an inflammatory model, also reported that TnC mediates synthesis of proinflammatory cytokines in the TLR4 pathway through post-transcriptional control on the micro-RNA level (Piccinini and Midwood, 2012). Mapping of the binding site of TnC showed that this molecule has direct and cooperative interaction with TLR4, but the same binding site was identified as a conserved inflammatory epitope in related proteins (Zuliani-Alvarez et al., 2017), thus confirming that TnC is a part of the TLR4 signaling cascade.

### Migration of Newborn Cells

After proliferation and survival, newborn cells at the stage of neuroblasts migrate to their final destinations. Besides the fact that astrocytes secrete growth factors and cytokines (Figure 3), those within the SVZ, RMS and OB express TnC throughout postnatal life, while migrating neuroblasts in the early postnatal subepidermal zone are also enclosed by a TnC-rich layer (Gates et al., 1995; Peretto et al., 2005). This suggests that TnC may play a regulatory role in tangential migration of neuroblasts, which could be attributed to its ability to form repellent interactions with other cell types (Husmann et al., 1995). Nevertheless, when this hypothesis was tested *in vivo* on TnC deficient mice the chain organization of the migratory pathway was unrelated to TnC deficiency (de Chevigny et al., 2006). In addition, in the SVZ explants culture there was no detectable difference in the rate of migratory neuroblasts between wild-type and TnC deficient mice.

In the SVZ of both postnatal and adult mice neuroblasts interact and modify the surrounding ECM by expressing matrix metalloproteinases (MMP), proteolytic enzymes that use components of ECM as substrates (Bovetti et al., 2007). TnC and other ECM components have been shown to influence neuronal migration in other brain regions through the proteolytic action of MMP (Murase and Horwitz, 2002). It has been reported that TnC is involved in cell migration through the activation of c-Jun N-terminal kinase, a member of the MAPK family, which further on modulates the expression and activity of MMP-9 (Cai et al., 2017). Another study confirmed the involvement of TnC in Wnt signaling (Figure 2), responsible for maintaining the stem cell pool and suppressing aberrant differentiation (Hendaoui et al., 2014).

*In vitro* migratory assays showed that TnC inhibits the migration of oligodendrocyte progenitor cells by inhibiting Wnt signaling (Kakinuma et al., 2004), which is in congruence with previous *in vivo* research evaluating the migratory activity of oligodendrocyte precursors in TnC deficient mice (Garcion et al., 2001). On the other hand, another study showed that TnC acts in a dose dependent way to promote the migration of bone marrow stem cells (BMSC) (Ding et al., 2018). Namely, when different concentrations of TnC are added to the medium where murine stem cells are seeded, high concentrations of TnC promote cellular migration. Additionally, it has been suggested that TnC can bind to TLR4 expressed on BMSC, and activate downstream signaling through MAPK, protein kinase B and Wnt signaling pathway. However, further studies are needed to unravel the role of TnC in cellular migration *in vivo*.

### Functional Integration of New Neurons

A critical factor for the selection process during the maturation of newborn neurons might be the rate at which newborn neurons are synaptically recruited, resulting in a better chance to survive. The functional importance of newborn neurons relies on their physiological properties. Namely, high excitability of newborn neurons when compared to mature cells, allows them to be more sensitive to synaptic plasticity.

Regulation of synaptic integration of adult-born neurons is shaped by actions of microglia through synaptogenesis and pruning, modulation of perisynaptic structures, and regulation of spine structure and synaptic transmission (Ekdahl, 2012). Microglia depletion in adult mice results in fewer spines with mushroom morphology, leading to overall reduced spine volume, and weaker excitatory synapses in the OB (Wallace et al., 2020). Synaptic transmission may occur in the perisomatic environment undergoing inactivation, degradation or activation of the ECM through the action of MMP-9, a molecule already confirmed to be involved in migration and differentiation of adult neural progenitors in the SVZ (Barkho et al., 2008). Another mechanism of microglial regulation of neuronal activity through remodeling of dendritic spine morphology, including size, shape and motility (Tremblay and Majewska, 2011), results in alterations in actin filaments (Fortin et al., 2012).

In the adult hippocampus, glutamatergic synapses onto newborn cells are characterized by an increased long-term potentiation (LTP) with a decreased induction threshold (Lledo et al., 2006). This was confirmed with single cell recordings in the hippocampal slices of adult rats, where immature granule cells in the DG were found to have lower LTP threshold compared to more mature neurons (Wang et al., 2000). Adult-born olfactory interneurons undergo different synaptic modifications compared with pre-existing mature interneurons (Nissant et al., 2009). A transient expression of LTP, and post-tetanic potentiation, were found exclusively in adult-born granule cells, not in pre-existing ones, making newborn granule cells particularly sensitive to synaptic plasticity. Thus, potentiation of the synaptic strength onto granule cells could increase feedforward inhibition onto olfactory bulb interneuron outputs, promoting efficient coding of information (Rinberg and Gelperin, 2006). Therefore, in both neurogenic regions, the ability of newborn neurons to balance excitatory/inhibitory inputs and outputs is crucial for their integration in existing circuits.

TnC has a prominent role in synaptic functions (Strekalova et al., 2002) and modulation of cellular behavior, since it is involved in the induction of LTP, possibly through the modulation of L-type voltage-dependent Ca^2+^ channels (Evers et al., 2002). It has also been reported that TnC has a prominent role in fine tuning of the balance between excitation and inhibition (Stamenkovic et al., 2017b). Namely, it was shown in TnC-deficient mice that the exposure to enriched environment (EE) induces lower expression of excitatory markers and a higher density of inhibitory terminals as compared to wild-type mice. An *in vitro* study in a three-dimensional nanofiber gel with a TnC derived peptide, showed extensive neurite outgrowth and increased expression of neuronal marker when compared to two-dimensional cultures (Sever et al., 2018). It is thus, plausible to emphasize that TnC may play an indirect role in neuronal differentiation and synaptic integration.

The effects of tenascin C on the above cellular processes (depicted in sections “Cell Proliferation,” “Survival of Newborn Cells,” and “Functional Integration of New Neurons”) are summed up in Table 1.

**TABLE 1:** Effects of Tenascin C on processes of proliferation, survival, migration and differentiation.

	**Effect**	**Species**	**Tissue**	**Age**	**References**
Proliferation	Increased	Mouse	SVZ	P0–P17	Garcion et al., 2001
	Decreased		Spinal cord	E14.5	Karus et al., 2011
	No effect		SVZ	3–5 m; N/A	Kazanis et al., 2007; Ding et al., 2018
Survival	Increased	Mouse	BMSC	N/A	Ding et al., 2018
Migration	Increased	Mouse	BMSC	N/A	Ding et al., 2018
	Inhibited	Mouse, rat	OG culture	P0, P2, E16	Garcion et al., 2001; Kakinuma et al., 2004
Differentiation	Suppressed	Rat, mouse	OG culture, whisker follicle	P0, P2; E10.5;	Garcion et al., 2004; Garwood et al., 2004; Czopka et al., 2010;
				N/A	Hendaoui et al., 2014
	Increased	Human	MSC	N/A	Tsai et al., 2014

*SVZ, subventricular zone; BMSC, bone marrow stem cells; OG, oligodendrocyte; MSC, mesenchymal stem cells; N/A, Not Applicable.*

## Importance of Adult Neurogenesis

Adult neurogenesis is a process considered as a type of cellular plasticity, an important mechanism for the regeneration of the CNS. The fact that the birth of new neurons in the adult rodent brain is conserved in the OB and the hippocampus, structures with high degree of structural and functional plasticity that are involved in storage and encoding of the sensory/memory information, qualifies these neurogenic brain areas for important roles in the physiological adaptation to new stimuli. A number of computational studies suggest theoretical roles of adult hippocampal neurogenesis, such as the increase of hippocampal memory capacity (Becker, 2005), reduction of interference between new and old memories, encoding of new memories (Wiskott et al., 2006), and the encoding of time in memories (Aimone et al., 2009). OB neurogenesis has not been as extensively studied computationally as hippocampal neurogenesis, but an *in vivo* study suggested that new neurons in their critical period of integration are required for the encoding of learning of odor related experience (Forest et al., 2019).

Impact of adult neurogenesis on cognitive functions is a matter of great complexity that needs to take a variety of factors into consideration, along with their interconnection and interplay. Moreover, all the functions of the hippocampus and the OB should be considered, hence a term of neurogenic niche has been introduced in order to explain the downstream influence of neurogenesis on behavior (Eisch and Petrik, 2012). This hypothesis could be supported by behavioral studies, that suggested a possible role of adult hippocampal neurogenesis in pattern separation (Clelland et al., 2009) and in memory consolidation (Kitamura et al., 2009). Moreover, manipulation of sensory input by odor deprivation or enrichment caused a decrease or increase, respectively, in survival of newborn interneurons (Bovetti et al., 2009). Another study that used odor enrichment as a paradigm, showed that treatment of mice with different fragrances resulted in an increased tyrosine-hydroxylase positive dopaminergic cell population, without changes in calretinin- and calbindin-positive neurons (Bonzano et al., 2014).

## Modulation of Adult Neurogenesis in Health and Disease

Dynamic regulation of different stages of adult neurogenesis in the hippocampus and the OB, including proliferation, survival, migration and integration, is under control of both intrinsic and extrinsic factors (Table 2). Environmental stimuli through exposure to an EE contributes to the survival of new granule neurons in the SGZ, without affecting the SVZ (Brown et al., 2003). Physical activity such as running, increases cell proliferation and survival of newborn neurons in the SGZ (Van Praag et al., 2005). On the other hand, enriched odor exposure increases proliferation in the SVZ, while the neurogenesis in the SGZ remains unaffected (Rochefort et al., 2002). Moreover, odor enrichment drives increased integration of newborn dopaminergic neurons (Bonzano et al., 2014).

**TABLE 2:** The effect of different factors on the processes of neurogenesis.

**Factor**	**Effect**	
	***SGZ***	***SVZ***
Enriched environment	↑ Survival	/
	Brown et al., 2003	
Physical excersice	↑ Proliferation	/
	Van Praag et al., 2005	
Odor enrichment	/	↑ Proliferation, migration, differentiation
		Rochefort et al., 2002
Age	↓ Proliferation	↓ Proliferation
	↓ Differentiation	Enwere et al., 2004
	Kuhn et al., 1996	
Stroke, ischemia	↑ Proliferation	↑ Proliferation
	↓ Survival	Sekeljic et al., 2012
	Takasawa et al., 2002	

Local environment, although providing signals for proper cellular development in physiological conditions, has a crucial role in keeping tissue homeostasis after injury or in pathological conditions. In the hippocampus of rats after focal cerebral ischemia an increased number of proliferating cells has been reported, but on the other hand, survival of newborn neurons has been reduced (Takasawa et al., 2002). In the experimental model of global cerebral ischemia, neurogenesis persists in the SVZ up to 1 year after the insult (Sekeljic et al., 2012). In fact, this study documented an increased number of proliferating cells and colocalization of markers of microglial activation and neurons. A proposed explanation delt with a beneficial role of microglia in chronic postischemic phase, supported by the findings of Ziv and colleagues, who suggested the microglia-T cell crosstalk to be a promoter for cell proliferation in the SVZ (Ziv et al., 2006). The same study has also put immune control over maintenance of adult neurogenesis in context of EE, suggesting that T cells are required for spatial learning and memory.

EE has been shown beneficial for many animal models of CNS disorders, such as Alzheimer’s and Parkinson’s disease, epilepsy or stroke (Young et al., 1999; Bezard et al., 2003; Jankowsky et al., 2005). Since NSC represent a constant source of cellular material for regenerative processes in the brain after injury, enhanced neurogenesis after exposure to EE could be additionally beneficial for disorders characterized by a reduced cell number.

It has been shown that aging has a detrimental effect on neurogenesis, with a decreasing rate of neurogenesis in later stages of life (Kuhn et al., 1996; Enwere et al., 2004). The process of aging does not only affect stem cells, but also their microenvironment. Namely, with the accumulation of stress-induced damage, such as induced by reactive oxygen species, local signaling pathways become dysregulated. Since decreased neurogenesis occurs in neurodegenerative disorders such as Alzheimer’s disease and depression (Rodríguez and Verkhratsky, 2011), while increased neurogenesis occurs in epilepsy (Jessberger and Parent, 2015), it can be concluded that this process is only beneficial within a physiologically adaptive range. Beyond a critical level of neurogenesis, the networks experience noise as a consequence of overexcitability. Considering all the conditions, it is not yet clear whether disrupted neurogenesis has a causative role in these disorders or a symptomatic one. A balance between the degenerative processes and the control of inflammation with neurogenesis could contribute to survival after global ischemia or in Alzheimer’s type dementia.

Thanks to the pleiotropic role of TnC in the CNS diseases, such as tumors, vascular and neurodegenerative diseases, this glycoprotein may be a candidate for clinical application (Hanmin et al., 2020). TnC has been recognized as another molecule involved in chronic inflammation in Alzheimer’s disease since its gene transcription is significantly increased in both cultured microglia after amyloid β (Aβ) peptide challenge, as well as in the brain of Alzheimer’s disease mouse model. In addition, TnC deficient mice have reduced proinflammatory but enhanced anti-inflammatory activity (Xie et al., 2013). TnC is upregulated in many human pathologies, and although it has been most extensively studied in the context of cancer, its immunomodulatory role also associates it with inflammatory diseases (Marzeda and Midwood, 2018). In adult human brains of AD patients, TnC was detected in diffused extracellular deposits in cortical gray matter, surrounding cored Aβ plaques (Mi et al., 2016). In addition, TnC plaques were associated with reactive astrocytes, microglia and Tau containing neurites. Furthermore, TnC was reported as a plasma biomarker of AD, since it is significantly increased in blood of AD patients (Soares et al., 2012). The beneficial effect of TnC on Alzheimer’s disease pathogenesis implicates this ECM glycoprotein as a new therapeutic target.

## Conclusion

As discussed here, TnC is considered as an important molecule for tissue repair and regeneration by participating in intracellular pathways that can lead to cell proliferation, survival and motility. Further studies need to integrate the knowledge about the role of TnC in adult neurogenic niches. Better understanding of the ECM signaling in the niche of the adult CNS will have significant implications for regenerative therapies. Strategies to enhance repair by endogenous stem cells or to replace lost cells by transplantation of exogenous stem cells could be improved by manipulations that mimic niche signals and therefore promote stem cell survival, proliferation and differentiation.

## Author Contributions

MT, PA, and VS were engaged in manuscript conceptualization. PA provided resources. MT was engaged in writing original draft preparation. PA and VS did writing—review and editing. All authors contributed to the article and approved the submitted version.

## Conflict of Interest

The authors declare that the research was conducted in the absence of any commercial or financial relationships that could be construed as a potential conflict of interest.
